# Application of Multimedia Networks in Business English Teaching in Vocational College

**DOI:** 10.1155/2021/5519472

**Published:** 2021-04-29

**Authors:** Xuexia Cheng, Kuifen Liu

**Affiliations:** International Business Department, Shandong Vocational College of Economics and Business, Weicheng, Weifang 261011, Shandong, China

## Abstract

To better meet the needs of economic restructuring and industrial development in China, educators in vocational colleges have to find new approaches to narrow the gaps between the updated requirements from the employers for business English majors and the vocational college education reality. Under this circumstance, a tentative study was carried out with the aids of multimedia to help the educators remove obstacles blocking achieving their educational aim, which is cultivating the graduates who are qualified for the social requirement. This study mainly discussed how effective the multimedia networks can help the business English majors in vocational colleges to enrich their work experience and enhance their practical English ability, computer skills, communication skills, and cooperation skills comprehensively. It aimed at exploring the ways of helping the business English majors in vocational colleges to gain work experience and improve their practical English skills, computer skills, communication skills, and cooperation skills with the aid of multimedia networks. An experimental teaching program was designed under the guidelines of a task-based teaching approach and constructive learning theory. The program includes four teaching models, which are in-class learning and field preparation, mock practice, in-field learning and field education, and learning reflection. All learning and field practices are delivered online facilitated by multimedia networks. One hundred and forty sophomores majoring in business English are selected as participants of the program. Data of students' confidence in all five monitored essential abilities are collected before and after the learning procedure through questionnaires, and students' feedbacks are collected through interviews. The statistical results show that multimedia networks can help students improve their overall competence, especially in gaining work experience and practical English skills. Moreover, adopting multimedia networks in teaching can provide more internship opportunities, enrich teaching scenarios, and prolong net teaching hours, which forms a preferred learning environment and provides better learning outcomes. It could also be used to assist communication and cooperation trainings.

## 1. Introduction

### 1.1. Background

Vocational colleges account for almost half of the advanced education in China, and the scale of vocational education is still increasing. Nevertheless, many of the graduates from the vocational colleges could not meet their employers' expectation. In fact, technology revolution and industrial transformation have generated higher demands on vocational college graduates, which lead to an acute structural imbalance between the expected skill sets and the actual competency of the new graduates.

To better meet the needs of economic restructuring and industrial development, many vocational colleges would send surveys about their education quality to employers, graduated students, and current students, and adjust the education plan for current students according to the survey responses. The survey conducted by Cheng Xuexia and the Business English Teaching and Research Section (2019) [1] shows four prominent inconsistency between the needs of labor market and the competency of fresh graduates from Business English majors in Shandong Vocational College of Economics and Business. First of all, students do not have sufficient field practice opportunities to accumulate practical skills of international trade. Secondly, in spite of having all required computer certificates, the English major graduates cannot fulfill their work via computer satisfactorily. Similarly, although the business English majors own several English certificates, their English skills are insufficient to deal with practical work. Last but not the least, these fresh graduates do not have adequate interpersonal skills, including cooperation or communication skills.

The lack of field education is one of the main causes for the abovementioned problems. For a long time, it has been a great challenge for vocational college students to find internship due to the limitation of the education system and government policies. It is even harder for business English majors to gain work experience as very few international trade companies offer field internship opportunities to vocational college students who are considered as uncompetitive and inexperienced.

The authors believe that adopting multimedia kits for teaching can help improve students' competence to the greatest extent—it would not only increase field practice opportunities but also enrich contents of field practice and improve teaching efficiency.

### 1.2. Conceptual Framework

In the past two decades, a clear shift in language-learning theory and research has led to a desire for more authentic communication in the classroom [2–6]. As a response to this call, learner-centered task-based teaching theory was developed for instructing learners of all proficiency levels in a variety of languages [5, 7, 8]. Constructivism is a theory about how people learn and acquire language by interacting with others [3].

#### 1.2.1. Task-Based Teaching Approach

Long [9] defines good tasks as “the hundred and one things people do in everyday life, at work, at play, and in between.” He points out that tasks given to students should come from the reality, which is authentic. Nunan [10] further elaborates good tasks as the sorts of activities that individuals usually do outside the classroom. He believes that good learning happens in the field, not in the classroom. Willis [11] emphasizes that good tasks should have two characteristics which are naturalness and worthwhile engagement. He believes tasks given by teachers should come naturally at that moment, which is proper and fit to students' learning; meanwhile, it should be worth practicing. Proponents of task-based teaching insist that the content of language learning must be relevant to all participants and learners should be involved in the planning, implementation, and evaluation of their instruction.

The traditional teaching methods are teacher centered, lecture dominated, and classroom based. In this teaching system, it is common for students to sit and listen to the lecturers in classroom, with very limited hands-on practice opportunity. When it comes to learning tasks, they are paper-based in general and usually generated from teachers' fabrication. The authors believe that, in order to help increase students' competence, it is important to shift the traditional teaching model to a student-centered, task-based, and field-based model. In the research program, teaching was largely put in the field and students became the center of the learning process with the help of the multimedia network. Meanwhile, tasks are naturally generated from a real working scene in the international business field, which are authentic and suitable for business English majors.

#### 1.2.2. Constructive Learning Theory

Constructivist theory sees knowledge as reorganization and reconstruction of experience that cannot be taught because it is unique for every individual [12]. Knowledge is not passively received but built up by the cognitive subject, and learning is an active construction based on the prior knowledge [13]. In the view of constructivists, learning needs not only the stimulation of the external environment but also learners' independent construction [14]. They believe students' learning is a multidimensional interaction among students, teachers, and the environment. The meaning is not given to learners, but is constructed by them according to how much their understanding is currently organized [15]. Krashen [16] holds the view that language learning should be a process of acquisition that takes place in a natural context instead of a process of learning language consciously. Knowledge is not obtained through rigid teaching, but with the help of others in a certain situation and through the means of meaning construction [17].

Dussault et al. [18] find there is a significant positive correlation between teaching efficacy and the effect of the application of multimedia in classroom teaching. The use of multimedia networks in teaching helps improve the original teaching model by adopting the constructive learning theory. It is believed that multimedia networks can not only create a fruitful and vivid external learning environment for students but also elicit students' passion of learning and continuously promote the process of inner knowledge construction [19]. In the research program, teachers used multimedia networks to form a multidimensional environment, which not only helps students become more qualified for real-life work and jobs but also enables students to be more confident and active to engage in the interactive activities.

The application of multimedia networks becomes even more significant under the COVID-19 pandemic. In this circumstance, all courses are taught online, which leaves no place for teachers to make face-to-face contact with their students. Neither could the students communicate with their classmates nor the external world face to face. Applying multimedia networks in teaching can compensate this disadvantage by integrating audio, video, images, animation, and text together on the teaching platform, which helps create a more intuitive, vivid, and lively virtual communication environment for the learners to interact with each other, with their teachers and the external world.

### 1.3. Empirical Evidence

Many attempts have been made on the application of multimedia networks in teaching. Hao [20] proposed an intelligent network teaching system model based on deep learning speech enhancement algorithm and robust expression positioning to recognize the students' general expressions in multimedia English teaching more accurately. Yu [21] created a multimedia and computer-network-aided classroom teaching model for college English and American literature course. Abdulrahaman et al. [6] provided a systematic review of studies on the use of multimedia networks in education to determine the extent to which multimedia has been successful in improving both teaching and learning. Oyeleye et al. [22] furthered the relative research to the tertiary education and illustrated multimedia technology utilization as correlates of lecturers' teaching effectiveness in colleges of education. Some virtual internship software and platforms have been developed to make up for the deficiency of internship posts and field practice opportunities. For instance, Li and Song [23] designed long-distance multimedia teaching system based on virtual reality. It can be used to make up for the gap between the needs of internship and the posts available. Such a virtual system relieves the stress of college English teachers and students and provides the students with more field-work-like scenes and they can simulate tasks in the real world. Yet, doing simulated tasks is still different from doing real field job. The desire to find chances to do the real international trade in field to gain the experience remains there.

More research studies focus on the theory construction and the advantages and disadvantages of applying multimedia networks in English teaching [23, 24]. Among them, the dominant theories are task-based learning theory and constructivist theory. The common acknowledged advantage of multimedia networks is that they facilitate the teaching of culture by providing immediate, ongoing contact with native L2 speakers [24]. Meanwhile, Cononelos [24] believes that networks can bring students and native speakers together to share information, negotiate meaning, and develop strategies for successful, authentic communication.

### 1.4. Aims of the Study

This study attempts to answer the following question: How effectively can the multimedia networks help the business English majors in vocational colleges to enrich their work experience and enhance their practical English ability, computer skills, communication skills, and cooperation skills comprehensively?

## 2. Methods

### 2.1. Teaching Program Design

There are four teaching modules in the program, including product exhibition, business relationship establishment, factory tour, and business negotiation, which form an essential series of the international trade procedure. Due to the outbreak of COVID-19, all lessons are carried out online, mainly on the Smart Teaching Platform. Meanwhile, students are unable to practice their knowledge in field in person as most companies suspended their operation. Nevertheless, to cope with the pandemic, many international trades are transferred from in-person activities to online ones, which offers students extra practical opportunities. Under this circumstance, the research team designed an experimental teaching program based on the multimedia networks, which was student centered, task based, and field based. In the program, learning mainly happens in the field and tasks are generated from real working posts. Each participant in the program would have a unique education plan and have a chance to gain and practice their knowledge in real working field through multimedia networks. It is believed that this teaching program can help improve the four primary deficiencies identified in the previous survey.

The core of this program is field education. Two online exhibition platforms, Online Canton Fair (from June 15 to 24, 2020) and Alibaba International Online Trade Show (from June 8 to 28, 2020), were selected as platforms to carry out field education, for the reason that their operation and business activities perfectly match with students' learning content. The research team reached a field education agreement with several manufacturers where business English students could perform their live broadcast as interns to get hands-on experiences. Students could find other companies as field placement if they could and would adhere to the requirements of epidemic prevention and control.

Learning in field has three stages: field broadcast experience, mock practice, and hands-on field practice. On the first stage, students can shadow the experienced employees in the international trade field. On these platforms, every participant in the exhibition would have a live streaming chat room for their company where they conduct live broadcast with all kinds of multimedia technologies to the public. When they are offline, their recorded live streaming can be continuously replayed in their chat room. This arrangement gives not only those attendees but also the students an opportunity to review their performance whenever and wherever they want. Students can learn from the live broadcast and borrow their work experience to improve and perfect their own work. On the second stage, students can practice their prepared materials on other teaching platforms such as the Smart Teaching System and QQ Group Classroom before they showcase to the audience. After presenting the mock broadcast on the Smart Teaching Platform, students will get comment from their partners, teachers, and field instructors to revise their performance. After the preparation, students can move to the third stage: to work in the field as interns. The research team, together with field work instructors from manufacturing companies, assigned remote field tasks to students and supervised the whole procedure. Students were expected to practice all four learning modules in their field education. During the program, students had access to background information of four manufacturing companies together with details of their products manifested through multimedia networks.

It was expected that students would strengthen their insufficient abilities by actively engaging in these field work, and receive valuable feedback from the research team and field instructors on the online teaching platform. For instance, in the process of product displays and negotiation, students were expected to gain more hands-on experience by doing live broadcast with graphs, videos, PowerPoint slides, and whiteboards, as well as making phone calls and writing business letters. As for English skills, students could practice useful language expressions used in the international business procedure. Meanwhile, to attract more visitors to their chat rooms and establish new business relationships, students were expected to make every endeavor to plan, design, and polish their courseware on computer, which gave them the opportunity to practice their computer skills. Moreover, such kind of complex tasks can barely be carried out by a single student without cooperation or communication with both the internal and external team. Thus, cooperation and communication skills would be developed correspondingly.

The detailed teaching program design is as follows (in Figure 1).

### 2.2. In-Class Learning and Field Preparation

Four sections, including language expression, multimedia skills, company-specific information such as products and company culture, and international business and trade knowledge and skills, are covered by in-class learning and field preparation. Language expression could be learned from textbooks and the smart teaching platform, as well as the experienced instructor in the field. Multimedia skills could be learned through the smart teaching platform, the Internet, and textbooks. Company-specific information, including products and company culture, is available on the smart teaching platform. International business and trade knowledge and skills could be learned from textbooks and field instructors as well.

### 2.3. Mock Practice

Before acting as an intern demonstrator in the field, students have a mock practice opportunity to rehearse and present their prepared work on the smart teaching platform. Students can improve their work with comments and suggestions gained from their teachers, field instructors, and classmates.

### 2.4. In-Field Learning and Field Education

Product exhibition: this section has four subtasks: (1) create PowerPoint slides for the product exhibition, (2) prepare auxiliary material for online live broadcast, (3) deliver live broadcast online, (4) and interact with visitors online.

Business relationship establishment: this section includes two subtasks: (1) reach out to customers who left their electronic business cards during the exhibition and (2) establish business relationship through multiple ways, including making phone calls, composing business letters, and through other media.

Factory tour: this is the third section of in-field learning and field education. Three tasks are included. (1) prepare for an online factory tour, including the language, related background information, and other techniques which can make the tour more impressive, (2) deliver a factory tour, and (3) keep in touch with customers who are interested with the products and supply them with a variety of information.

Business negotiation: this is the last section of this teaching model. Four subtasks include (1) prepare relative material for online negotiation, (2) know about the negotiation counterparts, (3) negotiate with counterparts online and reach a win-win situation, and (4) be aware of the desire and floor price of the negotiation counterparts, and meet the counterparts' requirements to the maximum extent on the basis of profit maximization of the presented company.

### 2.5. Learning Reflection

Learners reflect and improve their field work based on the actual effects of their field performance before representing to the public.

### 2.6. Survey Design

The survey in this study was designed by the research team led by Cheng Xuexia. It includes means of questionnaires and interviews. The pretest questionnaire and interview were delivered to the employers, the graduates, and current students. The posttest questionnaire was delivered only to the 140 current students who are the subjects of the study because only the 140 current students took part in the experiment. The questionnaires are composed of mainly multiple choices and several open-ended questions, both of which focus on the gap between the employment needs and the graduates/current students' ability. The interview was designed to gain more insights which may not be covered by the questionnaires.

The questionnaires were first carried out in the 2019 fall semester, in which five crucial concerns within students' performance were found (as shown in Tables 1–3). This series of questionnaires not only serve as one of the intermediate causes of launching this study and the experimental teaching program but also provide the pretest statistics. The posttest questionnaire was delivered to current students who were selected as participants of this program only. The same questions asked in the pretest questionnaire were asked again.

The posttest interview started with an open-ended question “How do you feel about this new education experience?” Based on students' responses, several follow-up questions would be asked to provide more details to supplement the quantitative findings in the questionnaire. Some of these questions include “What impressed you the most about the online field practice?” and “What influence did it take to you about your expression in English, computer skills, international trade experience, and cooperation ability?”

### 2.7. The Subjects

All 140 sophomores majoring in business English from Shandong Vocational College of Economics and Business were selected as participants of the experiment. All of them had finished international trade courses, acquired basic practical skills, and owned basic computer skills.

Demographic data of the subjects, such as age, gender, and birthplace, are also collected. In this study, all participants are at the age of 18 and 19. About 77% (108/140) of them are female, and 23% (32/140) are male. Around 82% (115/140) of the participants are local students from Shandong Province, and 18% (25/140) of them are from other provinces. All students are admitted through the national university entrance examination (Gaokao), which gives them similar learning background and study experience.

### 2.8. Data Collection

The questionnaire was delivered to all 140 participants in the study, and the interview was delivered to 16 students with random sampling. All 140 questionnaire responses and 16 interview samples were collected back. All data were collected through the face-to-face method by the author and her research team. The author supervised the whole research process to make sure that all staff would follow the same procedure and standards during the study and all subjects have the same understanding of every question asked and respond to the questionnaire and interview consistently within the data collection process.

### 2.9. Analytic Strategy

Statistical analyses were processed under SPSS (Statistical Package for the Social Science Version 26.0). Chi-square (McNemar's test) was adopted as a matched pair test to obtain comparable results for checking the same subjects in the pretest and posttest. The frequency of negative and positive responses in the questionnaire was tested.

## 3. Result

The statistical results (Pearson Chi-Square) are as follows (in Table 4).

The comparison statistic results shown in Table 4 demonstrate the differences in students' responses between the pretest and posttest figure. In general, students reported less worry in all five aspects after joining in the teaching program. Three aspects of students' confidence level have a less than or equal to 10% increase, including communication skills (7.2%, from 45.7% to 52.9%), computer skills (9.3%, from 40.0% to 49.3%), and cooperation skills (10%, from 50.7% to 60.7%). Other two aspects have a more notable increase, including self-confidence in English proficiency at work (16.5%, from 32.1% to 48.6%) and work experience (22.1%, from 24.3% to 46.4%). Pearson chi-square is calculated under *df* = 3, 95% confidence interval. The standard *p* value of English proficiency at work and work experience is less than 0.05, while the standard *p* value for other three variables is greater than 0.05.

As for the interview, students have a positive attitude towards the experimental teaching program in general and have more confidence in all five abilities trained in the program. Students believe that the multimedia networks work well as teaching instruments, especially in learning practical computer skills and reducing the fear of participating in group conversation and teamwork. During the program, many participants see the value of field practice and notice that English, as well as specialized knowledge learned in class is, to some extent, is different from the one normally used in field. Detailed quotes are included in the following discussion.

## 4. Discussion

The questionnaire contains five examined aspects, including the confidence level of computer skills, English proficiency, work experience, communication skills, and cooperation skills. By attending the experimental teaching program, students' self-confidence in all five aspects has increased in varying degrees, which indicates the positive impact made by this teaching program in general. In terms of students' confidence in computer proficiency (*I can use the computer to fulfill the work satisfactorily*), although it increases from 40.0% to 49.3%, yet, the *p* value equals 0.118, which is greater than the 0.05 significance level, under *df* = 3, 95% confidence interval. Hence, the observed chi-square is not significantly different from the expectation. Similarly, for students' confidence in communication (*I can communicate with colleagues, managers, and customers confidently and successfully*) and cooperation skills (*I can cooperate with partners efficiently and smoothly)*, the statistical results indicate that no significant changes have taken place (*p*=0.232 > 0.05, *p*=0.92 > 0.05, respectively). Therefore, although positive impacts have been made on students' computer skills, communication skills, and cooperation skills to some extent, shown by the increasing number of *yes* given by students in the posttest questionnaire, we cannot say that significant changes have taken place statistically.

As for English proficiency at work (*I can use English appropriately or confidently to deal with practical work)* and work experience *(I have adequate work experience)*, the statistical results (*p*=0.005 > 0.05, *p*=0.001 > 0.05, respectively) illustrate that the significant differences exist—students have a statistically significant increase and gain in their English proficiency at work and work experience by attending the designed teaching program.

The biggest difference between the traditional teaching model and the experimental one is that the former one does not include field practice. In other words, before joining the experimental teaching program, students had no access to work experience and practical English. On the contrary, the other three monitored aspects, including cooperation skills, communication skills, and computer skills, can be trained in the traditional teaching model to some extent. This could explain why students' confidence in English proficiency at work and work experience has significant improvement while the other three do not.

Three findings could be drawn from the chart and the abovementioned analysis, which show how effectively the multimedia teaching kit and field-centered teaching program can affect students' performance. First of all, although students' self-confidence in all five aspects has increased in varying degrees by attending the teaching program, their relative position in the sequence remain the same. Secondly, students' self-confidence in gaining work experience has the greatest increase (22%) among all five tested aspects; however, it is still ranked as the least confident item. Thirdly, work experience and English proficiency at work are ranked as the most and second unconfident items by students before the program; yet, it has the first and second greatest increase in the posttest.

As discussed, most students speak highly of each addressed ability, as well as the teaching program, in the follow-up interview. One of the typical responses is that *“I think many of us, just like me, had no faith in this program at the beginning. I was astonished that the program was so great after attending it…*.*”*

Some students go to details about why they like the program. *“Well, I like this semester's teaching. The most important gain is that I have confidence in myself now. I found that I can deal with the real tasks with my English and I know how to further improve it now. I am happy about it.”*

“The lack of field work experience had been confusing me. But, I now know about what it is like, to engage in the international business trade, at least to some degree, by means of the multimedia network. After tries both on the Online Canton Fair and Alibaba Online Trade Show, I feel assured that I have experienced it.”

*“Indeed, tasks in field are quite different from the artificial ones in the classrooms. They are neither so difficult nor so easy, just like what the fable The Little Horse Crosses the River says.”* He further explains, *“I think everyone has his own study pace. Tasks in field are quite flexible in the teamwork. We will only be assigned tasks that are fit for us. That is why I feel comfortable about it.”*

Dissatisfaction does exist, but is occasional. One student reports that his English proficiency and computer skills are not capable of keeping up with the work pace during the program. Other dissatisfaction is due to teaching-irrelative issues, such as Internet failure. For instance, one student reports *“I live in the countryside where Wi-Fi connection is weak. I lost connection with the Internet quite often, like for every 15 minutes.”* Two other students have similar problems with him that they missed a lot of chances to keep up with their classmates and failed to engage in activities. Other eight students report that they do not have computers; therefore, they also have to fulfill tasks on their smart phones, which is inconvenient.

In the interview, students were also asked about how they felt about comprehensively involving a multimedia kit into their study. Several respondents give different views about the effect of multimedia networks. For instance, one student reports that combining a multimedia kit and field work makes personalized study viable. In the traditional class model, one instructor is responsible for around 30 students. In this situation, everyone studies in the same classroom at the same time and follows one teacher only, where conducting individualized teaching is infeasible. Therefore, everyone studies in the same pace and does the same tasks with the course going on. Now, with the help of multimedia networks, instructors can arrange individual meeting with students at different time periods without letting other students wait, which is more productive and convenient.

Another student reports that *“Although we lost the chances to go back to the college classroom, yet multimedia networks made up the loss and offered us a more luxuriant one under the advice and guide of our teachers.”* When being asked about what the “luxuriant one” refers to, he elaborates that *“study becomes more interesting on the Internet where I can approach to abundance of challenging scenarios and practice different ways of reaching potential business partners.”*

As reported, the application of multimedia networks provides students the opportunity of field practice during the COVID-19 pandemic where tasks are authentic and more varied compared with the old ones, which makes students more involved into the learning process. Surprisingly, several students express that multimedia networks help them overcome the fear of communication and cooperation. *“Meanwhile, it is not so scary to communicate. Quite opposite, I can enjoy a lot of pleasure in communication and cooperation. After all, we can get in touch with each other through multimedia networks, which supply a lot of convenience and keep a lot of embarrassment away from us.” “I was originally afraid and reluctant to communicate with people. It is even harder for me to speak to a stranger. But, in field practice, I found it is a must. No communication, no customers from the trade show. So, it forced me to speak up ……. Basically, I watched how my supervisor does it through recorded videos and copied it at the beginning, when I had to introduce our products in the trade show……. At least, I am not afraid of communicating through video chat now.”*

It is interesting to see that multimedia networks as a supplement way of communication and cooperation work effectively. The research team thinks that thanks to multimedia networks, students can avoid physical interaction when communicating and can fully express themselves with aids from the multimedia.

## 5. Conclusions

Four conclusions could be drawn from this study. First of all, multimedia networks, especially when combined with field practice, can help business English majors improve their overall competence. Among all five monitored aspects, work experience and practical English are the two with significant improvement. Secondly, the application of multimedia networks provides a significant number of internship opportunities and enriches teaching scenarios. In this circumstance, students have more choices and would be able to apply their acquired knowledge to practice comprehensively. Thirdly, using multimedia networks as a teaching kit prolongs online teaching hours, which enables individualized teaching. Together with field practice, lecturers and tutors could provide fitted knowledge and tasks to students based on their study pace. Last but not the least, multimedia networks provide multi-interactive approaches which facilitate communication and cooperation among students. Teamwork and communication training based on multimedia networks could be designed and delivered to students needed. All in all, the novelty of this study is that the multimedia network is introduced to the tertiary business English teaching and a practical approach has been proposed to help relieve the challenge in tertiary business English teaching: the chances to get the field work experience.

## 6. Limitation and Implication

Firstly, the duration of the experiment is limited. In only four weeks, four main tasks are checked due to the late start of the online field activities. Secondly, due to the COVID-19 pandemic, all in-person field practices were suspended, which forced all students to participate in online field practice. Consequently, there was no controlled group. The comparison of the research items only existed between before and after receiving remote field practice. Thirdly, the subjects are limited to current students. Data from the employer side and graduate side are not collected in the posttest research.

In the future research, we will further investigate the proposed model using other databases, collect data and comments from employers and graduates who used to participate in online teaching program, and take their feedback into consideration. Moreover, longer experiment period and bigger sample size with both a controlled group and experimental group in non-English majors are suggested in the future research.

How much multimedia networks can devote to college English teaching will ultimately depend on teachers. Application of multimedia networks is just one of the many valuable resources available for learner-centered college business English instruction. The ways in which teachers integrate multimedia network services with other language-learning activities will be instrumental in deciding the long-term value of the multimedia networks in college business English education.

## Figures and Tables

**Figure 1:** The program design.

**Table 1:** Survey result from the 122 employers.

In your point of view, what is/are the main problem(s) for business English major graduates?	Frequency of yes	Total respondents	Percentage of yes
They lack field experience	109	122	89.34
They cannot use English appropriately or confidently to deal with practical work	63	122	51.64
They can communicate with colleagues, managers, and customers confidently and successfully	54	122	44.26
They need more practice in order to cooperate with partners efficiently and smoothly	52	122	42.62
They cannot use the computer to fulfill my work satisfactorily	89	122	72.95

**Table 2:** Survey result from the 566 graduates.

In your point of view, what troubles you the most in your first job?	Frequency of yes	Total respondents	Percentage of yes
I do not have enough field experience	235	566	41.52
I cannot use English appropriately or confidently to deal with practical work	227	566	40.11
I can communicate with colleagues, managers, and customers confidently and successfully	221	566	39.05
I cannot cooperate with partners efficiently and smoothly	198	566	34.98
I cannot use the computer to fulfill my work satisfactorily	378	566	66.78

**Table 3:** Survey result from the 140 current students.

In your point of view of your future career, what would be the main problem(s) that worries/worry you the most?	Frequency of yes	Total respondents	Percentage of yes (%)
I lack field work experience	106	140	75.71
I cannot use English appropriately or confidently to deal with practical work	95	140	67.86
I can communicate with colleagues, managers, and customers confidently and successfully	76	140	54.29
I cannot cooperate with partners efficiently and smoothly	69	140	49.29
I cannot use the computer to fulfill my work satisfactorily	84	140	60.00

**Table 4:** Paired comparison between pre- and postexperiment.

Select all statements that you feel comfortable about, in view of your future job	Pre-/posttest	Frequency of yes/no	Total responses		Value	df	Progressive significance (2 sided)
I can use computer to fulfill my work satisfactorily	Pretest	56/84	140	Pearson chi-square	280	3	0.118
	Posttest	69/71					
I can communicate with colleagues, managers, and customers confidently and successfully	Pretest	64/76	140		280	3	0.232
	Posttest	74/66					
I can use English appropriately or confidently to deal with practical work	Pretest	45/95	140		280	3	0.005
	Posttest	68/72					
I have adequate work experience	Pretest	34/106	140		280	3	0.000
	Posttest	65/75					
I can cooperate with partners efficiently and smoothly	Pretest	71/69	140		280	3	0.092
	Posttest	85/55					

## Data Availability

The data used to support the findings of this study are available from the corresponding author upon request.
